# Research on the Influence of Sports and Nutrition Matching on Improving Students' Physique Based on Intelligent Sensor

**DOI:** 10.1155/2021/3556131

**Published:** 2021-12-31

**Authors:** Yejin Wu, Fucai Zhang

**Affiliations:** School of Physical Education and Health, LinYi University, LinYi, Shandong 276000, China

## Abstract

With the continuous development of social economy, students' learning is paid more and more attention, but at the same time, their physical condition also deserves attention. In view of these problems and limitations, this paper is based on intelligent sensors, which is different from the traditional physical education teaching, adopts the corresponding prescription for sports teaching, combines teaching with fun for the corresponding health intervention, and realizes the two-way dimensional analysis of compound sports prescription through comprehensive nutrition collocation, so as to improve students' physical and mental health, in order to improve students' physical fitness. The simulation results show that the intelligent sensor is effective, which can improve the systematicness and scientificity of students' participation in exercise in sports activities and improve students' learning and physical fitness.

## 1. Introduction

With the continuous development of social economy, students' physical condition and learning situation have attracted more and more attention from society and families [1, 2]. More families pay more attention to academic performance and ignore physical exercise, which often leads to a lack of physical fitness [3, 4]. It is worth noting that students are the future of the country, and their health determines the long-term development of the nation and the economic revitalization of the country [5, 6]. Because of this, students' physical fitness should receive more attention. For students' physical health guidance, it is mainly carried out by guiding and heuristic strategies, which is not only an attempt of practical education, but also an important direction of participation. Compared with foreign practice, China's intervention for students is relatively less and the frequency is not enough [7, 8].

The continuous development of economy and society has promoted the improvement of people's material living standards, but excessive intake of eating habits and diet will lead to physical obesity, especially for young students [9, 10]. Therefore, scientific exercise and healthy nutrition are needed to ensure the balance of students' physique and prevent and solve the corresponding obesity problem. The government and families also regulate and guide students to exercise a healthy lifestyle through various forms, and give corresponding guidance, in order to improve the physical quality of young students, but these studies are still lacking and insufficient. For example, they cannot accurately grasp the physical problems of all students, because everyone's physical conditions are different and cannot be generalized. It cannot be simply used with the same sports and the same nutrition [11, 12].

In view of these deficiencies and needs, this paper introduces intelligent sensors, collects the current situation of physical education teaching, integrates the factors of health reform, uses corresponding prescriptions for sports teaching, and uses nutrition collocation to realize the two-way dimensional analysis of compound sports prescriptions, so as to improve students' physical and mental health, in order to improve students' physical fitness.

## 2. Relationship between Sports, Nutrition, and Immunity

### 2.1. Sports and Immunity

For immunity, it is an important component of human body function and an important barrier to protect body health. Good immunity is the guarantee to ensure that the body adapts to various environments. When the human body carries out sports or physical exercise, the human body's immunity is adjusted. Through the change of antibody, it is enough to resist the body's bad cells, make the body adapt to this environment, and guide the whole body's physique to improve. However, it should be noted that sports need to pay attention to the control of quantity. Appropriate sports are conducive to the improvement of body immunity, but excessive and high-intensity sports may be counterproductive. Long-term sports will consume people's body skills, and a large number of substances will continue to emerge. These substances will destroy the body's function and affect immune cells, reducing the immunity of human body. Therefore, in general, for sports, select appropriate and reasonable sports methods according to the individual's own situation to ensure the effective amount of exercise, which can not only achieve the purpose of physical exercise but also improve the immunity of human body [13–15].

### 2.2. Protein Nutrition and Immunity

For the human body, the protein and vitamins in the body have an impact on the function of the body's immunity, so as to have a certain impact on people's normal activities.

Nutrients such as protein or vitamins in the body will affect the body's immune function, which in turn affects the body's normal activities and exercise capabilities. Protein is one of the important elements of nutrients required by the human body. Insufficient protein intake will lead to a decrease in the number of related cells and phagocytes in the human body, which will reduce the function and ability of cytokines. Too little secretion of synthetic substances will lead to human diseases. The increase in probability affects the normal functioning and actions of the human body. For example, human fitness athletes control the intake of protein foods when they lose weight. During the process of weight loss, phagocytes are also reduced, which affects the healthy operation of the overall function. When performing protein control experiments in animals, the experimental mice with long-term low protein intake are exercised. After a period of time, the experimental mice will develop ketemia, and the immune function of the experimental mice will decline through inspection and development, which will eventually lead to the immune organs atrophy and aging. Performing normal activities under the condition of insufficient protein intake will lead to insufficient energy supply to the immune system, coupled with the body's demand for protein for exercise, the immune function will be affected by the lack of nutrition, and the immune system will be destroyed. After the conclusion of the influence of protein intake on the immune system is reached, in order to further confirm the direct impact of protein, the protein intake of experimental mice can be increased. After a few weeks, the cell function and response ability of experimental mice are observed, and the function of phagocytes is gradually improved, which further indicates that the intake of protein nutrition will directly affect the function of the body's immune system.

For protein, in fact, it is an important nutrient required by the human body. If the human body lacks enough protein, it will further affect the body and affect normal physical activities. For example, for sports athletes, if the intake of protein is reduced, it will affect the normal operation of the whole body function and even lead to the atrophy of corresponding body immune organs. Relevant studies have shown that the intake of protein nutrition will directly affect the immune system of human body [16–18].

## 3. Research Method

### 3.1. Experimental Research Method

First, set the corresponding smart sensor. You can set the data transmission delay of the terminal request location and the server base station location to *D*, and the clock deviation of the two locations is set to Δ*t*. The server base station receives the corresponding data at T2 and T3, respectively and replies the response data to the request terminal. After the data request terminal receives the corresponding data, you can use formula (1) to carry out quantitative calculation.

The deviation calculated by each request terminal can be corrected according to the corresponding atomic clock to realize the time synchronization between the data request and the data server.

(1) $$\begin{array}{c} \left\{\begin{array}{c} T_{2}=T_{1}+d+\Delta t\\ T_{4}=T_{3}+d-\Delta t \end{array}\right.\Rightarrow \left\{\begin{array}{c} d=\frac{\left(T_{2}-T_{1}\right)+\left(T_{4}-T_{3}\right)}{2},\\ \Delta t=\frac{\left(T_{2}-T_{1}\right)-\left(T_{4}-T_{3}\right)}{2}. \end{array}\right. \end{array}$$

On this basis, the data request terminal applies for corresponding data, including the number of terminal nodes, the period of time slot, the start and end time of time slot, and other corresponding metadata information. These parameters are initialized and analyzed by the data request terminal.

After receiving the corresponding data from the data server, the data request terminal determines that the specific time of the data request terminal is unknown according to the data information, so the corresponding configuration can be completed according to the static time slot. The specific calculation is shown in formula (2). When the data request terminal needs data transmission, data transmission is carried out.

(2) $$\begin{array}{c} t_{i}=t_{0}+\left(i-1\right)\times 2l+k\times T,\;k\in \left\{0,1,\ldots \right\}. \end{array}$$

It should be noted that when the data requesting terminal retransmits data in the time slot of server retransmission, first, retransmission Part 1 is retransmitted, and the time at this time can be calculated by formula (3); when retransmission Part 1 does not receive the response data from the data server, it enters retransmission Part 2. At this time, the retransmission time slot can be calculated by formula (4). When retransmission Part 2 does not receive the response data, it enters retransmission Part 3 for continuous transmission similar to 1 and 2. At this time, the retransmission time slot can be calculated by formula (5). However, if the response data from the data server is still not received, the terminal requests the node to stop the continuous transmission of data, enter the planting state, and wait for the next cycle of the administrator.

(3) $$\begin{array}{c} t_{1}=t_{0}+\left(n+r_{1}\right)\times 2l,\;r_{1}\in \left\{0,1,\ldots ,\frac{n}{5}\right\}, \end{array}$$

(4) $$\begin{array}{c} t_{2}=t_{0}+\left(\frac{6n}{5}+r_{2}\right)\times 2l,\;r_{2}\in \left\{0,1,\ldots ,\frac{n}{25}\right\}, \end{array}$$

(5) $$\begin{array}{c} t_{3}=t_{0}+\left(\frac{31n}{25}+r_{3}\right)\times 2l,\;r_{3}\in \left\{0,1,\ldots ,\frac{n}{125}\right\}. \end{array}$$

When the data terminal node encounters emergency data transmission, it first needs to obtain the authentication of the data server. It can communicate with the terminal through the data server, so as to allocate the shadow time slot. The specific calculation is shown in formula (6).

During data transmission, the data request terminal transmits data in the shadow time slot of the data server.

(6) $$\begin{array}{c} t_{j}=t_{0}+\left(2j-1\right)\times l+t\times k,\;k\in \left\{1,2,\ldots \right\}. \end{array}$$

This paper selects the corresponding student groups for research, one class as the experimental class and the other class as the corresponding verification class, as shown in Figure 1.

Before the corresponding intervention in physical education teaching, distinguish the specialties and interests of the corresponding students according to the actual requirements, such as giving the courses with the corresponding selection resources (gymnastics, basketball, table tennis, and martial arts) as the main body, integrating the corresponding quality physical exercise and physical games, and building an appropriate physical exercise mode and an excess of a certain amount of physical exercise mode. Fully mobilize the enthusiasm and independent selectivity of students and physical education teachers.

According to the existing research, we choose to change from three aspects: trend, generalization, and integration, so as to ensure the combination of theory and practice in physical education, realize the learning of theoretical knowledge in physical education, consolidate skills in practical exercise, and improve physical fitness. In these two stages or time periods, students can realize the combination of theory and practice and gradually develop their interests [19, 20]. In the actual exercise process, it can be distinguished according to the actual needs and conditions.

1. Firstly, the corresponding comprehensive physical fitness test is carried out to test the strength, speed, and endurance, respectively. The teachers arrange the frequency and intensity of follow-up physical exercise according to different physique.
2. In the experiment, learning and teaching are carried out according to different actual needs and venue needs, according to the corresponding plan, and the theoretical teaching is carried out in the form of new media such as audio and video, so as to improve the interest and novelty of physical education teaching.

### 3.2. Investigation Method

The research method used in this paper is shown in Figure 2. From the results, it can be seen that the corresponding effective rate can be obtained in multiple measurements before and after the intervention. The average effective rate of the data used for quantitative analysis is higher than 86%, which meets the requirements of statistics.

In the actual investigation and research, the corresponding teachers, students, and parents were selected for unified discussion and interview, and the key groups were contacted by means of mobile phone, e-mail, and letters to ensure the process and effect of the experiment.

On this basis, the authors also visited many sports theory experts and physical education teachers to conduct corresponding consultation and analysis from the current situation of physical fitness and exercise.

### 3.3. Programming

Intelligent sensors are used, through the use of appropriate teaching methods to improve students' sports habits, at the same time, with comprehensive nutrition matching, so as to improve students' physical health level.

According to the data analysis and comparison of the corresponding classes, the same PE teachers are selected. The experiment is carried out without the knowledge of the students.

For PE teachers' lesson preparation, it is carried out in the way of seeking common ground while reserving differences through collective lesson preparation, so as to realize the completion of PE structured teaching. According to the statistics of weekly physical education classes, the heart rate is monitored by intelligent equipment to collect data and master the intensity of exercise in real time. The two classes in the experimental comparison adopt the same class hours, and the content of physical education curriculum is also the same.

## 4. Simulation Experiment and Analysis

### 4.1. Experimental Implementation

Stretch before sports by setting up warm-up exercises, such as sit-ups and rope skipping.

The use of intelligent sensors to monitor heart rate can realize the real-time monitoring of exercise frequency and intensity, enable students to participate in sports more actively and independently, and ensure that the exercise reaches a certain load but does not exceed a certain amount.

In the later stage of exercise, the data after exercise are collected through the final exercise, such as sit-ups.

#### 4.1.1. Evaluation of Intervention Effect of Physical Education and Healthy Exercise Prescription on Students' Physique

*(1) Influence of sports and health exercise prescription on students' physical quality*. As shown in Figure 3, through the intervention after the combination of sports and nutrition, the excellent rate of physical quality in the experimental group was significantly higher, increased by 8%, the good rate increased by about 20%, and the unqualified rate decreased. From the next point of view, the comprehensive combination of sports and nutrition had an obvious good effect on the improvement of students' physical quality and ensured that students had good exercise habits, improving students' physical quality.

The results after the comprehensive intervention are shown in Figure 4. The students in the experimental group are more active in spirit and have higher enthusiasm, especially compared with the nonintervention group. At the same time, the sense of quietness and fatigue have changed, indicating that the students are actively participating in physical exercise, but they still have a certain degree of fatigue psychologically, which is worthy of attention.

*(2) Effects of physical education and healthy exercise prescription on students' health knowledge, belief, and behavior*. From the results in Figure 5, it can be seen that after intervention in the five groups of A, B, C, D, and E, students' scores in sports theory knowledge are more obvious, increasing by about 50%, and participation in healthy behaviors has even increased. About 53%. The simulation results show that the smart sensor is effective and can effectively monitor.

*(3) Effects of sports and health exercise prescription on students' social adaptability and mental health*. Physical education activity is a group activity to complete the teaching task through the interactive behavior of teaching, learning, and practice between teachers and students and students.

#### 4.1.2. Evaluation of the Intervention Process of Physical Education and Health Exercise Prescription Education

During and after the intervention, the researchers, teachers, and students in the experimental group evaluated the selection of teaching contents, teaching methods, teachers' teaching ability, and effect. Nutrition is not only the material basis of growth and development, but also an important factor to improve health and physique. In recent years, with the continuous improvement of living standards, people's physical quality does not increase infinitely with the improvement of living standards. Nowadays, the physical health of middle school students is facing the dual challenges of malnutrition and malnutrition.

*(1) Expert teacher's evaluation of intervention in the education process*. During the intervention process, three senior teachers (education inspectors) from the experimental school were hired to quantify the teaching situation of the experimental teachers. Specific teaching evaluation is mainly based on teachers' preclass preparation, teaching goals, completion of tasks, application of teaching strategies, students' learning status, ability to deal with emergencies or special situations in class, and summary after class. In the “Evaluation Criteria” column, the full score for each item is 5 points, for a total of 100 points. From the comprehensive score after the end of the experiment, the total average score of the experimental teachers is 88.85, and the score shows a trend of increasing from front to back. It shows that teachers' teaching ability is gradually improving, and they can be well qualified for intervention teaching work.

*(2) Students' evaluation of intervention in the education process*. After the experiment, the experimental group students fill in the “Comprehensive Evaluation Form of Physical Education and Health Education” to score the teaching ability and teaching situation of the experimental teachers. It mainly includes five items: teaching objectives, teaching content, teaching process and methods, basic teaching qualities, and immediate effects of teaching. The total score for each of the secondary indicators is 10 points, totaling UX points. The average score of experimental teachers is 87.42 points.

*(3) The relationship between teaching effect, teaching content, teaching method, and teacher's teaching ability*. In the “Sports and Health Education Evaluation Form,” students are asked to self-evaluate their achievements in physical education and mental health on a 100-point scale. The higher the score, the greater the gain. The significance of the differences in the scores of the students is tested in different experimental classes in the four aspects of their learning gains, teaching content, teaching methods, and teachers' teaching ability. The results showed that the scores of the 8 experimental classes in 4 aspects were not significantly different (*P* > 0.05). It shows that the level of the experimental teachers is quite equal, and the teacher's factor has little effect on the experimental results.

By analyzing the relationship between students' nutrition, harvest, and teaching content, multisource regression analysis is carried out. From the evaluation of teaching content (x1), teaching method (x2), and teaching ability (x3), as shown in Figure 6, it can be seen from the results that the equation can be fitted as *y* = 1.54 + 0.47 × 1 + 0.95 × 2 + 0.77 × 3, indicating that the three factors affect the teaching effect. At the same time, the higher the scores of the three factors, the greater the students' harvest. In addition, teaching methods and teaching ability have a great impact on teaching effect.

Nutrition is the material basis for growth and development, and it is also an important factor for improving health and improving physical fitness. With the continuous improvement of living standards in recent years, people's nutritional status and physical fitness have improved to a certain extent. However, people's physical fitness level does not increase indefinitely with the improvement of living standards. It usually has a rapid growth stage after basically satisfying people's living standards, and when it reaches a certain level, it is in a slow stage. If continuous supplementation of large amounts of nutrition leads to overnutrition, it will also lead to a decline in physical fitness; that is to say, malnutrition or excess will lead to reduced physical fitness. As the most important meal of the day, breakfast is of great significance to young people who are burdened with heavy academic pressure and are in a critical period of growth and development. However, among the students tested, there are still 15.42% of students who never eat breakfast or only eat breakfast 1–2 times a week, 2.68% of students never drink milk, and 3.20% of students never eat eggs. The positive adolescents in the vigorous growth and development period should consume 12% to 14% of their total energy every day, and more than half should be high-quality protein. These students who do not eat eggs and milk should obtain protein in their daily diet. Insufficient or poor quality may lead to retarded growth and weakened immunity. In severe cases, weight loss, short stature, anemia, delayed sexual development, and retarded mental development may occur. In addition to malnutrition, overnutrition is also an important factor leading to the decline of middle school students' physical fitness. The obesity rate of Chinese adolescents is increasing. The current obesity rate of urban boys is 14.2%, which has exceeded the 10% “safety threshold” announced by the World Health Organization. Among the students tested, 248 drank more than two bags of milk a day and 463 ate eggs every day, but 33% of these students still failed to pass the physical fitness test. Excessive nutritional conditions can sometimes inhibit health to a certain extent. Therefore, the physical health of middle school students nowadays is facing the double challenge of malnutrition and overnutrition.

### 4.2. Influence of Attitude on Physical Health of Middle School Students

Students' own attitude: with the continuous development of social economy, students' lifestyle has also changed, especially satisfied with the current situation, unwilling to exercise, and only willing to sit and indulge in mobile intelligent devices, which has a direct impact on teenagers' physical quality. At the same time, due to the few physical education courses offered in schools, most students are unwilling to take the initiative to participate but are greatly affected by their families. There are still many students willing to participate in sports to improve their cognition and physical quality. As the main body of the test, middle school students basically understand that the main purpose of participating in physical exercise is to strengthen their physical fitness and improve their physical health. With the development of the national fitness movement and the increasing importance of the school's physical health status of middle school students, it has promoted the enthusiasm of middle school students to participate in physical exercise, and the personal willingness of middle school students to enhance their physical fitness also directly affects the effect of exercise. Research shows that 88.27% of middle schools offer at least 1 to 2 physical education classes every week, mainly for students to exercise and improve their physical fitness. Most students expressed their willingness to participate in physical education classes. Only 0.84% of the students did not like to participate in physical education classes, and these students failed in the physical fitness test.

School attitude: the sports activities that the school should carry out include school sports, morning exercises, break exercises, and organized extracurricular activities. It is difficult for the amount of exercise of middle school students to meet the exercise intensity required by the growth and development of middle school students.

Parents' attitude: the large-scale emergence of the only child and the changes in family relations are also important factors affecting the physical health of middle school students.

There is a significant correlation between the number of physical exercises and the physical health of middle school students. The experiment shows that the less the number of physical exercises, the worse the physical health.

## 5. Conclusions

As China moves forward to become a sports power, students' physical health has become one of the directions paid more and more attention. Therefore, in view of these limitations, this paper introduces intelligent sensors to distinguish from traditional teaching, teach students according to their aptitude, formulate corresponding prescriptions for teaching intervention, and not only improve students' physical and mental health, but also improve students' physical quality. At the same time, it integrates nutrition collocation to realize the two-way dimensional analysis of compound sports prescription. Simulation experiments show that the intelligent sensor is effective and can improve students' sports level and physical quality.

## Figures and Tables

**Figure 1:** Statistics of the number of subjects.

**Figure 2:** List of basic information of each scale (questionnaire).

**Figure 3:** Comparison of physical fitness grades of middle school students after intervention and back test.

**Figure 4:** Comparison of physical exercise sensory changes of middle school students after intervention and back test.

**Figure 5:** Comparison of awareness rate of KAP questionnaire after intervention.

**Figure 6:** Correlation between variables in multiple regression analysis.

## Data Availability

Data sharing is not applicable to this article as no datasets were generated or analyzed during the current study.
